This article has been retracted.

# Construction of Mitochondrial Protection and Monitoring Model of Lon Protease Based on Machine Learning under Myocardial Ischemia Environment

**DOI:** 10.1155/2022/4805009

**Published:** 2022-10-08

**Authors:** Jinliang Wang, Yang Zhang, Haijiao Shi, Ying Yang, Shuai Wang, Fengrong Wang

**Affiliations:** ^1^Liaoning University of Traditional Chinese Medicine, Shenyang 110000, China; ^2^Shenyang Fourth People's Hospital of China Medical University, Shenyang 110000, China; ^3^Department of Cardiology, Affiliated Hospital of Liaoning University of Traditional Chinese Medicine, Shenyang 110000, China

## Abstract

The localization of a protein's submitochondrial structure is important for therapeutic design of associated disorders caused by mitochondrial abnormalities because many human diseases are directly tied to mitochondria. When Lon protease expression changes, glycolysis replaces respiratory metabolism in the cell, which is a common occurrence in cancer cells. The fact that protein formation is a dynamic research object makes it impossible to reproduce the unique living environment of proteins in an experimental setting, which surely makes it more challenging to determine protein function through experiments. This research suggests a model of Lon protease-based mitochondrial protection under myocardial ischemia based on ML (machine learning). To ensure the balance of all submitochondrial proteins, the data set is processed using a random oversampling method, each overlapping fixed-length subsequence that is created from the protein sequence functions as a channel in the convolution layer. The results demonstrate that applying the oversampling strategy increases the ROC value by 17.6%-21.3%. Our prediction method is successful as evidenced by the fact that ML prediction outperforms the predictions of other conventional classifiers.

## 1. Introduction

Lon protease is an ATP-dependent serine protease, and it is also a member of ATPase protein family related to various cellular activities. It has a serine-lysine catalytic structure and can play an important role in degrading folding errors and damaging protein, maintaining the stability of intracellular environment and structure. Mitochondrial structure-function relationship is mainly regulated by molecules that regulate mitosis and fusion between mitochondria [1]. In cytoplasm, nucleus, and endoplasmic reticulum, the above proteins are usually degraded or eliminated by proteasome, while in mitochondria, lysosomes need to autophagy or degrade proteins, such as Lon protease, to complete this work, so as to maintain the mitochondrial homeostasis. Myocardial ischemia-reperfusion injury and diabetes consequences are both caused and developed in part by mitochondrial oxidative stress [2]. Numerous studies have demonstrated that Lon protease mediates the turnover of aberrant protein and short-lived protein. In addition, it rigorously detects the substrate during the enzymatic hydrolysis of protein and contributes to the determination of the intracellular protein life. Lon protease has been linked to a number of diseases, including lipid metabolic disorders, cancer, and ageing in recent years, according to an increasing number of studies.

As the energy factory of mitochondrial cells, it plays an important role in the life process of organism. Studies have shown that mitochondrial dysfunction is the potential mechanism of drug toxicity. Drugs directly or indirectly destroy mitochondrial structure and function, which can lead to mitochondrial toxicity, and may lead to target organ toxicity. As a heat shock protein, one of its main functions is protein quality control. In bacteria, the mutation of Lon protease showed abnormal protein degradation defects, which proved the role of Lon protease in protein quality control. In addition, Lon protease can also bind to DNA and affect DNA replication and gene expression. However, the activation of protease is not enough to degrade all the carbonyl protein accumulated in mitochondria, so Lon protease may be easily inactivated when oxidative stress increases, leading to mitochondrial dysfunction and nerve cell death. It was found that 90% of LONP1 exists in the mitochondrial matrix in soluble form, while 10% exists in the mitochondrial inner membrane. The division process prevents the abnormal elongation of mitochondria by splitting a single mitochondria into two independent daughter mitochondria. The research on crystal structure of Lon protease provides conditions and also lays a foundation for us to screen inhibitors and activators of Lon protease from natural products or synthetic small molecular compounds with high throughput and to develop drugs acting on Lon protease.

The function of mitochondria has drawn a lot of interest in the study of cancer mechanisms. In addition to performing oxidative phosphorylation, mitochondrial cells also produce heme protein, lipid, amino acids, and nuclear acids and take role in controlling the stability of the internal environment. Numerous human disorders, including Parkinson's syndrome, diabetes, and Alzheimer's disease, have direct links to mitochondria. Drug design for disorders similar to those caused by mitochondrial abnormalities can benefit from knowing where a protein's submitochondrial structure is located. Each subcellular coordinated the division of labor and worked together under the direction of genetic information, ultimately achieving the unity of the internal system of cells and the orderly progression of various life functions, such as metabolism and heredity. The subcellular localization prediction of Lon protease under myocardial ischemia was thoroughly studied in this paper based on ML (machine learning) method [3, 4] and support vector machine, in order to improve their current prediction quality and provide a practical, efficient, and affordable research method for proteomics.

Research innovation:

1. The method used in this research to extract protein features is based on self-cross covariance transformation and combines position correlation score matrix, pseudoamino acid composition, and dipeptide composition to address the issue of restricted single feature. Utilize the limit gradient hoist to screen out crucial characteristics and eliminate superfluous and pointless features
2. In this paper, ML correlation algorithm is used to analyze the trajectory of molecular dynamics simulation of Lon protease. Taking residues and protein as units, from the details, observe the influence of each residue site on the overall movement of protein

This paper is divided into five sections, and the specific arrangements are as follows.

The first section introduces the background work of the research. The second section mainly introduces the present situation of this research. In Section 3, a model of mitochondrial protection by Lon protease based on machine learning under myocardial ischemia is proposed. The fourth section verifies the performance of the model studied in this paper. The fifth section is the conclusion.

## 2. Related Work

### 2.1. Study on Mitochondrial Protease Correlation

Lon protease can degrade oxidized proteins in mitochondrial matrix, so it plays a key role in dealing with oxidative stress such as hypoxia or ischemia. The change of Lon protease expression leads to the change of cell metabolism, from respiratory metabolism to glycolysis, which usually occurs in cancer cells. Pomatto et al. demonstrated that LONP1 performed a crucial “scavenger” role in mitochondria, specifically destroying aberrant protein. In the same way, LONP2 performed a comparable function in the peroxisome [5]. According to Gong et al., acute stressors such as heat shock, serum hunger, and oxidative stress can cause LONP1 expression to be upregulated for a prolonged period of time, which is followed by an increase in aberrant protein clearance and cell survival rate [6]. According to research by Lee and Zhao, upregulation of LONP1 expression can reduce insulin resistance and treat type 2 diabetes whereas downregulation can disrupt insulin signal transduction and raise glucose allozyme levels [7].

The importance of mitochondrial fusion in heart development has been described by intrauterine death in the second trimester of pregnancy after Mfn1 and Mfn2 gene ablation. Andrianova et al. made a new discovery in the experimental results: mitochondrial fusion factor Mfn2 can interact with AMP-activated protein kinase to mediate cell survival under energy stress [8]. Babin et al.'s research on HL-1 cell line pointed out that Drp1 played an important role in the process of mitochondrial fragmentation, which was verified in mouse myocardial infarction model [9]. Mitochondrial-dependent protease not only has proteolytic activity but also plays a role of molecular chaperone, which promotes the assembly of protein complexes. When some sites of these proteases are mutated, the proteins in mitochondrial inner membrane cannot be transposed normally, and some subunits cannot be assembled normally, resulting in abnormal cell function. Jeannette used the third repetitive sequence of baculovirus inhibitor of apoptosis protein as affinity reagent and confirmed that the mature serine protease Omi/HtrA2 in mitochondria is protein and caspase activator that can directly bind to the third repetitive sequence of baculovirus inhibitor of apoptosis protein by elution, microsequence analysis, and spectral measurement [10].

### 2.2. Research Status of Bioinformatics

Biology and information industry complement each other, and the combination of them produces bioinformatics. It should be pointed out that at present, almost all these databases are free for academic research departments or personnel and can provide free downloads and other free services. Many of its research results can be industrialized quickly or immediately and become high-value products. This feature of bioinformatics is almost unique in many existing disciplines.

The ultimate goal of the study of protein is to understand its function and mechanism. Because protein formation is a dynamic research object, it cannot simulate the specific living environment of protein under experimental conditions, so it undoubtedly increases the difficulty of measuring protein function by experimental methods. Figaj et al. made use of bioinformatics methods to study and discuss it from various angles and achieved certain research results [11]. Osuagwu et al. put forward a protein function prediction model based on protein's block weight coding, which ignores protein-protein interaction and only starts from protein sequence, to solve the function prediction problem of protein without interaction partners [12].

The SubMito method was developed by Stocker et al. based on the characteristics of the protein sequence in order to identify and predict the location of the protein's submitochondria. SVM (support vector machine) localization and prediction model was established, and the overall prediction accuracy was 85.2% [13]. The broad properties of pseudoamino acid composition in protein omics were first proposed by Reunov et al., and since then, numerous methods of pseudoamino acid composition variants have proliferated [14]. Chou's pseudoamino acid composition was combined with evolutionary information, physical qualities, and chemical properties by Huang et al., who employed multicore SVM as a classifier and produced significant advancements in the localization of human proteins [15]. The gene expression profile data can be filtered to increase the prediction accuracy. Sharma et al. derived the evolutionary information from the location-specific score matrix. Without experimental annotation, this technique can increase the accuracy of protein prediction [16]. The ML approach based on omics data was partitioned by Niehaus et al. into a model using the closest neighbor technique [17]. Signal processing technology has its own special benefits in detecting this periodic feature buried in signals, as Yashas et al. noted that the function of protein may be manifested through a certain periodic energy distribution [18].

## 3. Methodology

### 3.1. Parameter Selection of Feature Extraction Method

Lon protease was first found in *Escherichia coli*. Later, it was found in many organisms, but the full-length crystal structure of protein has not been reported so far. Lon protease contains both ATPase and proteolytic enzyme activities in the same peptide chain. This structure is also found in HflB protease, but these two proteases are located on two different peptide chains in Clp protease family. Most studies think that Lon protease belongs to the family of heat shock proteins [19]. For example, in *Escherichia coli* and *Bacillus subtilis*, the expression of Lon protease gene is induced by high temperature.

Lon protease plays an important role in methylation-dependent cell cycle regulation. Lon protease may affect early cell replication and other processes by interacting with other protein. Upregulation of Lon protease can prevent the oxidative damage of protein and lipid, keep the balance of mitochondrial redox, reduce the level of mitochondrial complex I, and alleviate the heart injury. Besides regulating ATP-dependent protein degradation, Lon protease also has the function of molecular chaperone. Furthermore, Lon protease has the characteristic of binding to DNA [20]. Therefore, exploring a more efficient and sensitive method to explore the components and mechanism of mitochondrial dysfunction caused by traditional Chinese medicine can provide a reference for further understanding the toxicity of traditional Chinese medicine and provide a basis for guiding clinical safe drug use.

The localization prediction of Lon protease mitochondrion can be regarded as a multiclassification problem in ML. The first step of applying ML method is to transform protein sequence into feature vector, that is, feature extraction. This step is crucial, which determines the highest threshold that the model performance can reach. Amino acid composition information can reflect the physical and chemical properties of molecules. Protein located in the same subcellular position has similar amino acid composition information because it adapts to the same microenvironment. In the research, the protein sequence is often segmented, and then the amino acid information of each segment is calculated, and finally, the new vector is formed by recombination. Once the positioning of protein deviates, it will cause cell dysfunction and even cause many serious diseases such as cancer and Alzheimer's disease, which will have a significant impact on life. Therefore, the information of Lon protease subcellular localization can provide necessary help for the functional annotation of protein.

Protein is the main undertaker of life activities, and all life activities of organisms cannot be separated from protein. As a dynamic research object, the complete protein group still lacks effective research methods. It is not only necessary to predict the function of protein by calculation method but also has its theoretical basis. At present, although some prediction algorithms have high overall prediction accuracy, the prediction results are very unbalanced. The prediction accuracy of some functions is very high, while others are very low. Therefore, it is necessary to establish a standard and unified protein sequence database for a fair and just evaluation of protein function prediction algorithms.

GMM (Gaussian mixture model) is a widely used clustering algorithm. In essence, GMM is a mixed model. It measures things (data) by using Gaussian density function and decomposes things into multiple Gaussian density functions, that is to say, a set of data is fitted by multiple Gaussian models. Gaussian density function formula is as follows:

(1) $$\begin{array}{c} f\left(x\right)=\frac{1}{\sqrt{2\pi \sigma }}\exp\left(-\frac{{\left(x-\mu \right)}^{2}}{2\sigma^{2}}\right). \end{array}$$

In ML and statistics, EM (expectation maximization) algorithm is an iterative method, which is mainly used to find the maximum likelihood estimation or the maximum posterior probability of parameters in statistical models. That is, when these variables are known, the problem will be transformed into a simple problem, and the maximum likelihood solution will be obtained directly.

When the samples are nonlinearly divisible, a great idea of SVM is to use the concept of “kernel” and many kernel functions such as radial basis function, polynomial and multilayer perceptron to deal with nonlinear problems through projection transformation. Therefore, the optimization objective function after introducing kernel function is:

(2) $$\begin{array}{c} f\left(x\right)=\mathrm{sgn}\left(\overset{N}{\underset{i=1}{\sum }}a_{i}^{*}y_{i}K\left(x,x_{i}\right)+b^{*}\right), \end{array}$$

where *a*_*i*_^∗^, *K*(*x*, *x*_*i*_) represents Lagrange multiplier and kernel function, respectively.

For 2-dimensional or 3-dimensional data, the clustering results can be evaluated by visualization, but the visualization of high-dimensional data is difficult to realize. This paper chooses the S_Dbw method, which can be evaluated by two standards at the same time. When the data is completely separated, this item should be 0, that is, there is no data between different classes. Evaluation of intraclass indicators is mainly based on variance to evaluate the dispersion of intraclass data. The specific formula is as follows:

(3) $$\begin{array}{c} \text{Scat}\left(c\right)=\frac{1}{c}\overset{c}{\underset{i=1}{\sum }}\frac{\left|\sigma \left(v_{i}\right)\right|}{\sigma \left(s\right)}, \end{array}$$

where *c* represents the number of classes, *σ*(*v*_*i*_) calculates the variance of classes centered on *v*_*i*_, *s* represents the whole data set, and *σ*(*s*) calculates the variance of the whole data set.

RF (random forest) is to use Bootstrap sampling to get *k* sample data sets, train *k* classifiers, and then, vote for the majority of the results of multiple decision trees. It has good classification performance and accuracy and is robust to feature selection. Schematic diagram of RF classification is shown in Figure 1.

Firstly, the submitochondrial data set of protein is trained in *k* rounds to get {*h*_1_(*X*), *h*_2_(*X*), ⋯, *h*_*k*_(*X*)}, and then, the multiclassification model is constructed by voting method. Among them, the final classification decision is:

(4) $$\begin{array}{c} H\left(x\right)=\arg\underset{Y}{\max}\overset{k}{\underset{i=1}{\sum }}I\left(h_{i}\left(x\right)=Y\right). \end{array}$$

*Y* is the output variable, and decision tree *h*_*i*_ is a single decision tree (or objective function). By majority vote, the categorization is ultimately decided.

The description of metamorphosis *T* initially creates a substitute sequence by changing the original sequence. *T* has three features, including the frequency of dipeptide compositions from polar groups to neutral groups and from neutral groups to polar groups, as well as the frequency of dipeptide compositions from neutral groups to hydrophobic groups and from neutral groups to polar groups. The following defines a *T* descriptor:

(5) $$\begin{array}{c} T\left(r,s\right)=\frac{N\left(r,s\right)+N\left(s,r\right)}{N-1}, \end{array}$$

where *N*(*r*, *s*), *N*(*s*, *r*) is the frequency of dipeptide coded *rs*, *sr* and *N* is the sequence length.

When the training samples are nonlinear, a nonlinear function *ϕ* can map the training sample set to a high-dimensional linear feature space. In this linear space with infinite dimensions, the best classification hyperplane can be built, and the discriminant function of the classifier can then be obtained. The categorization hyperplane then becomes:

(6) $$\begin{array}{c} w\cdot \phi \left(x\right)+b=0. \end{array}$$

With the addition of the kernel function, SVM can now handle a large number of nonlinear problems without having to perform laborious nonlinear transformations on the samples in the input space. Instead, it uses the kernel function to map the samples to a high-dimensional linear space and create the ideal classification hyperplane, effectively resolving the “dimension disaster” issue.

### 3.2. Construction of Protection Model

Lon participates in the assembly of protein complex, but does not depend on its protease activity. Stress in endoplasmic reticulum can accumulate abnormal proteins in endoplasmic reticulum and damage mitochondrial function. Under the condition of glucose repression and amino acid starvation, these nucleosome proteins will be recruited into the nucleosome and recombined with other nucleosome constituent proteins. The dynamic localization of these proteins leads to mitochondrial nucleosome remodeling. This may be because the efficiency of Lon protease decreases with age, and a higher expression level is needed in order to maintain the same activity level as that in young cells. When mtDNA mutation accumulation reaches a certain threshold, it can lead to clinical symptoms of mitochondrial dysfunction-related diseases. Therefore, the lack of stress response ability of Lon protease may be a manifestation of the decrease of adaptability of cells during aging.

In addition, there are other ATP-dependent protease inhibitors in bacteria, such as RexB protein which inhibits Clp protease activity through unknown mechanisms. For example, the respiratory function of yeast Lon protease mutant is affected, and it cannot grow in nonfermentable carbon source medium. Moreover, the abnormal accumulation of mitochondrial protein leads to electron enrichment in mitochondrial matrix and loss of mitochondrial DNA function. The problem of mitochondrial localization prediction is essentially a multiclassification problem. Generally, training predictive classifiers is based on data sets with basically balanced sample distribution. There is another problem with the fused features, which may be high-dimensional or have redundancy and noise, which is not conducive to the training of the model. Removing irrelevant features can not only reduce the difficulty of learning tasks but also help alleviate the dimension disaster.

Mitochondria are important organelles in eukaryotic cells and participate in key physiological processes such as cell differentiation, cell information transmission, cell apoptosis, and growth. Enzymes have strict requirements on reaction conditions, such as pH value and temperature, which have specific limits. Exceeding the limits can cause denaturation and decomposition of enzyme proteins. Therefore, it is necessary to develop an automatic and reliable theoretical prediction method. So far, bioinformaticians and biochemists have developed many theoretical methods. However, the sequence alignment methods all rely on the protein sequences or structures with known functions. For protein which lacks sequence similarity or structure similarity with other protein, the existing methods are difficult to predict the functions of these unknown protein. Some proteins have the same domain, but they have completely different functions. All these problems have brought great difficulties and troubles to the existing methods of predicting the function of protein.

In recent years, some breakthroughs have been made in the research of Lon protease submitochondria localization, and some predictors have been developed. These predictors are all used to predict the submitochondrial position in the outer membrane, inner membrane, and matrix of mitochondria. Because of the limitation of the number of protein, the mitochondrial membrane gap is always excluded. Although these methods have achieved good performance, there are still some limitations. Based on this, this paper proposes a model of mitochondrial protection by Lon protease based on ML under myocardial ischemia, as shown in Figure 2.

Random oversampling method is used to process the data set to ensure the balance among all kinds of submitochondrial proteins. The protein sequence is cut into a plurality of overlapping fixed-length subsequences, and each subsequence serves as a channel in the convolution layer. Next, train a multichannel two-layer CNN (convective neural network) to learn advanced features in the sequence. Multichannel CNN is used to extract features from protein sequences and predict the results.

In order to fully consider the relationship between different features and find out more critical feature information for subcellular localization, attention mechanism is used to weight the fused features. The final output attention numerical matrix is calculated as follows:

(7) $$\begin{array}{c} \text{Attention}\left(Q,K,V\right)=\text{soft }\max\left(\frac{{QK}^{T}}{\sqrt{d_{k}}}\right)V. \end{array}$$

*V* represents weight value, *K* represents keyword, and *Q* represents query.

The values of independent variables and dependent variables of correlation are uncertain, and they can be interchanged. Correlation analysis is used in many research fields, including biology. It can measure the correlation between two or more variables. The ratio of covariance to standard deviation of two variables is used to reflect the linear correlation between two variables, usually expressed by the lowercase English letter *r*. The formula is as follows:

(8) $$\begin{array}{c} r=\frac{\sum_{i=1}^{n}\left(X_{i}-\bar{X}\right)\left(Y_{i}-\bar{Y}\right)}{\sqrt{\sum_{i=1}^{n}{\left(X_{i}-\bar{X}\right)}^{2}\sum_{i=1}^{n}{\left(Y_{i}-\bar{Y}\right)}^{2}}}, \end{array}$$

where *X*, *Y* represents two variables and *n* is the sample size. The greater the |*r*|, the greater the linear correlation between the two variables. *r* is regular, which means that there is a positive correlation between the two variables, and vice versa. When *r* = 0, it means that there is no linear correlation between the two variables.

We suggest a position-weighted amino acid component to extract the position information of residues near methylation sites such that the sequence information is not lost. For a sequence segment *p* containing 2*L* + 1 amino acid residues, we express the position information of amino acid *a*_*i*_(*i* = 1, 2, ⋯, 18) in the peptide segment *p* by the following equation:

(9) $$\begin{array}{c} C_{i}=\frac{1}{L\left(L+1\right)}\overset{L}{\underset{j=-L}{\sum }}x_{i,j}\left(j+\frac{\left|j\right|}{L}\right). \end{array}$$

In which *L* is the number of upstream residues or downstream residues on the symmetric peptide *p* from the central site, if *a*_*i*_ is the residue at the *j* position of the peptide *p*, then *x*_*i*,*j*_ = 1; otherwise, *x*_*i*,*j*_ = 0.

After feature transformation in convolution layer, the output feature map will be transferred to pool layer for feature selection and information filtering. Using pooling operation can eliminate irrelevant or unfavorable features without losing important information and reduce the complexity of model and calculation. Pool operation includes maximum pool and average pool.

(10) $$\begin{array}{c} h_{t}^{\left(2\right)}=\text{pool}\left(h_{i:n+i-1}^{\left(1\right)}\right). \end{array}$$

After a convolution and pooling operation, the potential feature vector is *H*^(2)^ = [*h*_1_^(2)^, *h*_2_^(2)^, ⋯, *h*_*l*−*b*+1_^(2)^], and then, the probability score (binary classification or multiclassification) is output through the fully connected network.

## 4. Experiment and Results

A computational model based on protein sequence must be built in order to perform exact positioning; hence, it is important to choose unbiased and representative benchmark data sets. The data sets used in this study are M317, M495, and M983, and each data set is broken down into three subregions: the inner membrane, the matrix, and the outer membrane. Few unknown proteins often have more than one known function companion protein. The known interacting protein in these instances, however, does not have the same functional type. When predicting a protein's secondary structure, sequence similarity of 30% indicates that the two sequences have the same folding structure; however, a sequence similarity of 40% indicates that the two sequences are not in the same subcellular location.

We use sliding window strategy to extract symmetric peptide segments centered on arginine and lysine from protein sequences to construct positive and negative sample data sets. The methylated skin segments of arginine and lysine labeled as “potential,” “probable,” or “by similarity” are excluded here. Arginine and lysine skin segments from the same protein in the positive sample without any methylation information are defined as negative samples. Finally, in order to ensure fair and objective results, we randomly select 90% of the data sets to build training sets and 10% to build independent test sets. In order to prevent the sampling deviation of the independent test set, the independent test set was sampled 10 times repeatedly, and the result of cross-validation in this paper is the average of 10 times.

In this paper, Pytorch backend is used to conduct all experiments on Nvidia Ge Force 2080TiGPU. Adam algorithm is used to optimize. The batch data size is set to 36, the iteration number is 200, and the fixed learning rate is 0.002. To avoid overfitting, we set the dropout ratio to 0.6. Firstly, we explored the performance of Ref [12], Ref [14], and the deep fusion evolutionary information method in this paper on two data sets, and the experimental results are shown in Table 1 and Table 2.

As can be seen from the table, the features extracted by different methods are integrated by the deep fusion evolutionary information framework in this paper, which can extract more abundant protein sequence information, and the prediction results are improved to different degrees compared with a single feature. Compared with the single special collection Ref [12] and Ref [14] in M495 data set, the overall actual accuracy of this method is 0.9553, which is 0.0913 and 0.0763 percentage points higher than that of Ref [12] and Ref [14], respectively. It can also be seen that the other four indexes of this method are better than only using a single feature.

The practical significance of residue clustering results is the conformational change of residues, that is, the change of spatial structure. The more clusters, the more conformational changes. The result of the conformational change of residues corresponds to the conformational distribution of each residue. According to the conformational distribution, the mutual information between every two residues is calculated to observe the correlation between residues. In order to understand the relationship between mutual information value and distance, we have drawn Figures 3 and 4.

Figure 3 shows the mutual information between every two residues in a scattered way. From the general trend, the farther the distance is, the smaller the mutual information between residues is. This also proves the rationality of this method.  Figure 4 shows that there are many pairs of residues with a distance of 25 to 95, and the mutual information values are all less than 0.05. Except for the very close mutual information, the mutual information between residues is mostly between 0 and 0.1.

The signal is divided into a number of wavelet coefficients via the wavelet transform. Different decomposition scales have varying outcomes when used to analyze protein sequences. A lengthy sequence cannot be broken down into its component parts on a tiny scale. We must select an appropriate decomposition scale in order to achieve the best prediction outcomes. The prediction outcomes of mitochondrial outer membrane and chloroplast inner capsule cavity are mostly explored here because this study seeks to increase the prediction quality of those two components.

Limited by the characteristics of wavelet decomposition, the analysis results of different decomposition levels are quite different. On the one hand, a large number of redundant data will be introduced when decomposing a short sequence; on the other hand, many details will be ignored when decomposing a small number of layers of a long sequence. We compare the data of 1-8 layers of wavelet decomposition to determine the optimal decomposition level. The results are shown in Figure 5.

Figure 5 shows that the fourth layer is the best decomposition layer for text selection since the total prediction accuracy rate obtained while decomposing to this layer is 93.323%, which is greater than the prediction success rate of the other layers. In order to verify the influence of random oversampling on the performance of the model, the receiver-operating characteristic curve is used to estimate the predictor. The multiclass ROC curves of two repeated experiments are shown in Figure 6.

Figure 6 shows a variety of ROC curves using oversampling method in the data set. It can be seen that the ROC value increased by 17.6%-21.3% after using the oversampling method. In this way, it is verified that the effect of adopting oversampling method is better than that of not adopting oversampling method, and the performance of the model can be improved. The ML prediction method constructed in this paper integrates two common classifiers. In order to verify the effectiveness of this integrated deep learning, we also use two basic classifiers for comparison. The results are shown in Figure 7.

To forecast the protein-protein interaction, we employ the integrated residual CNN. According on the experimental findings, this approach performs predictions better than SVM and XGBoost classifiers. Through layer-by-layer learning, ML prediction can mine the prospective feature data of protein interaction pairings, which fits the nonlinear relationship between sequence feature data and category labels well. This method's prediction accuracy is 94.28%. Our prediction method is successful as evidenced by the fact that ML prediction outperforms the predictions of other conventional classifiers.

## 5. Conclusion

As the energy factory of mitochondrial cells, it plays an important role in the life process of organism. The research on crystal structure of Lon protease provides conditions and also lays a foundation for us to screen inhibitors and activators of Lon protease from natural products or synthetic small molecular compounds with high throughput and to develop drugs acting on Lon protease. At present, although some prediction algorithms have high overall prediction accuracy, the prediction results are very unbalanced. Some functions have high prediction accuracy, while others are low. So, based on this, this paper proposes a model of mitochondrial protection by Lon protease based on ML under myocardial ischemia. In order to fully consider the relationship between different features and find out more critical feature information for subcellular localization, attention mechanism is used to weight the fused features. Compared with the single special collection methods in M495 data set, the overall actual accuracy of this method is 0.9553, which is 0.0913 and 0.0763 percentage points higher than other models, respectively. After using the oversampling method, the ROC value increased by 17.6%-21.3%. In this way, it is verified that the effect of adopting oversampling method is better than that of not adopting oversampling method, and the performance of the model can be improved.

## Figures and Tables

**Figure 1:** RF classification.

**Figure 2:** Schematic diagram of protection model construction.

**Figure 3:** Distance and mutual information diagram of conformational change of residues.

**Figure 4:** Distance of conformational change of residues and distribution of mutual information.

**Figure 5:** Prediction accuracy of different layers.

**Figure 6:** ROC curve of predictor in balanced data set.

**Figure 7:** Contrast result.

**Table 1:** Results of different feature extraction algorithms in M317 data set.

Evaluating indicator	Our	Ref [12]	Ref [14]
Average accuracy	0.9622	0.857	0.921
Overall positioning accuracy	0.9571	0.8553	0.9249
Overall accuracy rate	0.911	0.8533	0.8945

**Table 2:** Results of different feature extraction algorithms in M495 data set.

Evaluating indicator	Our	Ref [12]	Ref [14]
Average accuracy	0.973	0.8426	0.8768
Overall positioning accuracy	0.9553	0.871	0.9003
Overall accuracy rate	0.9553	0.864	0.879

## Data Availability

The data used to support the findings of this study are available from the corresponding author upon request.
